# Juvenile Delinquency from the Perspective of Socialization and Social Control

This article has been retracted.

**DOI:** 10.1155/2022/8657491

**Published:** 2022-10-10

**Authors:** Tingting Zhang

**Affiliations:** ^1^Guangdong University of Petrochemical Technology, Maoming 525000, Guangdong, China; ^2^Faculty of Law, Macao University of Science and Technology, Aomen, China

## Abstract

In recent years, the crime rate of minors in our country has risen steadily, laying a hidden danger for the harmonious and orderly development of the country and society. The healthy growth of teenagers is not only related to the harmony of a family and the future of a nation but also to the destiny of a country. Therefore, in order to ensure the healthy growth of young people and prevent juvenile delinquency, we should start with the causes of juvenile delinquency, identifying the core issues, so as to better study juvenile delinquency. In schools and families, strengthen the education of minors and guide them to develop positively. In terms of law, strengthen the supervision of minors to prevent them from breaking the law.

## 1. Introduction

The phenomenon of juvenile delinquency can be defined from multiple angles. In criminology, juvenile delinquency generally refers to the phenomenon in which people under 14 and under 25 are punished for breaking the law. Sociology focuses on the study of juvenile delinquency.

## 2. Youth Cybercrime

Compared with ordinary juvenile delinquency, the age structure of juvenile cybercrime groups tends to be younger. For one thing, this is due to the different ways of committing crime. The tool for juvenile cybercrime is the computer network, which greatly reduces the age limit in terms of physical strength and access to tools. For another thing, ordinary computer operation does not have high requirements from people, and the average elementary school students are fluent and skilled enough to operate it [1]. Young people lack self-control and cognition of their behavior; therefore, the scale of juvenile cybercrime has expanded rapidly. With the continuous development of the age of science and technology, computer applications are becoming more and more popular, and the scope of juvenile cybercrime has rapidly spread from the city to the countryside. In China, there are a large number of left-behind children in rural areas, and the intensity of education management is much lower than that in cities. As more and more rural left-behind youths come into contact with the Internet world, their lives are monotonous and lonely, which have changed dramatically [2]. Young children are more likely to be “abetted” by criminals when they make calls on the Internet and contact unsafe and unhealthy information, which leads to the continuous expansion of the scale of juvenile cybercrime.

## 3. The Causes of Youth Cybercrime

### 3.1. Weak Will and a Lack of the Ability to Identify Right from Wrong

As shown in Figure 1, when a person is in adolescence, he will be impulsive and self-willed because he lacks responsibility. In addition, their understanding of the law is far from normal. Teenagers have relatively weak willpower and are more prone to incitement by illegal information on the Internet [3]. Many criminals at home and abroad have pointed to immature young people, and the online platforms that young people often use are the worst-hit areas for bad information. However, due to their wrong understanding of new things, it is more likely to cause many serious consequences [4].

### 3.2. Insufficient Supervision of Families and Schools, Not Paying Attention to the Cultivation of Legal Awareness

A good family environment and strong school supervision are often the basis for avoiding youth cybercrime. However, in this regard, schools and society lack real supervision and supervision. In particular, there is still a considerable gap between the current requirements for school legal education and the new requirements for school legal education in the Internet age [5]. The school lacks legal educators who are proficient in both business and network technology, which means they cannot help young people understand the network in a timely manner, abandon uncivilized and unhealthy online activities, and stop online criminal activities in a timely manner. The lack of discipline and legal awareness will lead children to make illegal activities on the network.

### 3.3. The Uneven Network Environment and a Lack of a Strong Supervision System

The supervision system is a system formed by a series of legal provisions and various provisions promulgated by the state to supervise the state organs and their staff's compliance with laws and disciplines in state management activities [6]. The supervision system includes a wide range of content, including not only the legislative, administrative, and judicial supervision of state organs but also the supervision of political parties, the masses, and public opinion. Today's Internet is full of vulgar, bloody, and violent content, including reactionary and inciting speech that has penetrated from abroad. Due to a lack of self-control and the ability to distinguish right from wrong, our teenagers have become the most easily accepted objects of such bad information on the Internet [7]. Today, we have to think deeply about issues such as school violence, youth violent crimes, and youth online reactionary comments.

## 4. Prevention and Treatment of Youth Cybercrime

With the frequent occurrence of juvenile cybercrime, how to prevent and control juvenile cybercrime has become a major issue of concern to all walks of life [8]. The author analyzes the characteristics and causes of juvenile cybercrime and puts forward the following prevention and control measures, as shown in Figure 2.

### 4.1. Strengthening the Guidance Education for Young People and Cultivating Legal Awareness

For young people in a period of vague consciousness, their world outlook, values, and life views have not been fully established. Therefore, they need active and correct guidance and education from all walks of life [9]. Schools should develop specialized legal education to cultivate young people's good legal awareness and psychological quality and to eliminate the hidden dangers of crime. At the same time, young people should be educated in cybersecurity to increase their awareness and immunity against harmful information and cultivate their network behaviors and good network psychology [10].

### 4.2. Strengthening the Construction of Internet Culture and Creating a Good Network Environment for the Young People

Relevant departments should carry out “green network” activities for the whole society and prohibit users from posting vulgar, pornographic, violent, bloody, and other bad information on the network platform [11]. If any problems are found, the government will seize the illegal website and punish the relevant personnel. When departments are establishing a sound age classification system to prevent imperfect youths, they should also avoid premature contacting with inappropriate articles. Reasonable measures should be taken to prevent young people with improper concepts of right and wrong from being exposed to bad online information and provide them with a relatively good online environment [12].

### 4.3. Formulating Relevant Laws and Regulations to Combat Youth Cybercrime

The author believes that computer cybercrime, especially juvenile cybercrime, can be incorporated into the legislative focus in recent years. For one thing, a more comprehensive and scientific computer network legal system will be promulgated to form a set of reasonable and effective management systems to strengthen the management of cybercrime. For another thing, it is necessary to increase the crackdown on cybercrime against minors [13]. At present, laws and regulations are not enough to properly punish minors for cybercrime. Therefore, the author recommends that in order to prevent and control minors' cybercrime, the state should promulgate reasonable and perfect relevant network laws and regulations to increase the intensity of attacks on minors' cybercrime and maintain social stability.

## 5. Characteristics of the Times for Juvenile Delinquency

President Su of “*World Education Information*” pointed out the characteristics of the era of juvenile delinquency in our country during the interview.

### 5.1. Su Chunjing: The Current Situation of Juvenile Delinquency Is Mainly Manifested in the Following Six Points

First, the number of crimes has increased, and the environment is harsh. Juvenile delinquency almost involves the entire criminal field, among which theft, robbery, and provocations are the most common, especially new types of crimes such as online fraud and involvement in triad crimes. Secondly, the causes of crime are simple, which are sudden and blind. Due to lack of social experience and strong rebellious psychology, young people have poor self-control abilities and are prone to impulses [14]. Third, the crime committed is obviously younger. Since the 1990s, juvenile delinquency in my country has become significantly younger. The fourth is the occurrence of criminal methods towards high-tech crime. With the development and popularization of science and technology, the phenomenon of young people using high-tech or technological products to commit crimes is increasing [15]. Fifth, gang crime has increased, and the trend of grouping is obvious. Sixth, juvenile offenders are mostly children from divorced and poor families. In judicial practice, juvenile offenders have more children from divorced and poor families, who are generally low in education and weak in legal awareness [16].

### 5.2. Four Stages of Juvenile Delinquents' Growth Trajectory

The first is bad behavior. Juvenile delinquency often starts with low-level bad behaviors, including smoking, alcoholism, skipping classes, addiction to the Internet, participating in gambling, watching pornographic violence or reading materials, running away from home for no reason at night, running away from home, and so on. The second is illegal. Due to weak supervision or disobedience of the teacher's teaching, the seriousness of minor crimes has gradually increased, and there have been illegal acts such as fights, robberies, and theft. The third is crime. If a minor commits a crime, which cannot be corrected in time, he will constitute making mistakes [17]. The fourth is a serious crime. Criminology considers intentional killing, intentional injury to cause serious injury or death, rape, robbery, drug trafficking, arson, explosions, and poisoning as serious crimes. If minors do not repent after committing multiple crimes, they will most likely commit serious crimes in the end [18].

## 6. Research Situation of Youth Social Education at Home and Abroad

### 6.1. Development of Social Education of Young People Abroad

Before the 16th century, when society helped vulnerable groups, whether it was economic or material, the week would be divided into youth groups and adult groups. After the 16th century, people must not only serve the disadvantaged groups but also gradually extend the service to all children and adolescents [19]. Due to the early development and rich experience of Germany and the United States, the level of social education development is relatively high. For example, Germany clearly stipulates in the “*Juvenile Protection Law*” that children aged 4–18 must be systematically and comprehensively educated in health. The clear provisions of this law prompt German governments at all levels to attach importance to health education [20]. There are state institutions and many professional organizations in society.

Social education in Asia started late, and Japanese social education occupies an important position in their education system, which is closely related to the importance of the government. In the middle and late last century, the concept of lifelong education began to spread in the Japanese education community [21]. Therefore, more and more people of insight in Japan realize that social education and school education are inseparable for personal development.

### 6.2. Youth Social Education Development in Our Country

Compared with other countries in Asia, our country's social education is better, but compared with the old developed countries, there is still much room for improvement. From the perspective of historical and cultural processes, as early as China's primitive society, there has been a relevant social education [22]. The ancient Chinese peasant economy paid attention to learning and researching practical technologies, such as firewood and fire, Shennong farming education, and so on, which are social education of social education. In current society, the development of social education in Hong Kong, Shandong province, and other places is relatively prominent. For example, Hong Kong advocates a new social education model, with theory first. Therefore, in the study of social education theory, Hong Kong has strengthened its research on western successful models and regarded social workers as the main advocates of social education [23]. It opposes multiple educational models that use NGOs and social media as a means of publicity and education.

## 7. The Necessity of Social Work Intervention

### 7.1. Theoretical Aspects

From the perspective of China, its society is in a critical period of transformation. Social change conflicts with the individual's original three views, the formed way of thinking, and habitual behavior, which makes the socialization of adolescents endlessly difficult. Based on this background, more and more scholars regard youth social education as the main research object. Since reform and opening up, the current status of social education has improved significantly. The purpose of youth social education is to help them better integrate into social life. This requires that in the education of young people, it is necessary to ensure the improvement of adolescents' practical ability and the integrity of their socialization. At the same time, this kind of education should be combined with school classrooms and parent family education.

### 7.2. Practice

Judging from the time effect of the existing social work intervention in the social education for adolescents, social work can largely standardize works and promote the formation of the social education system.

As early as the second half of the last century, scholars in developed Western countries believed that social education was equivalent to social work. They consider that social education is “the science of social work.” Therefore, the essence of social education is that the target of social work is the youth group. The purpose is to let young people understand social work through social work methods. The goal and content of social work are to understand the true value of social work so that after learning social work, adolescents can use corresponding methods to analyze social behavior so as to achieve the purpose of learning about society, understanding society, and integrating into society. Therefore, social work and education are inseparable, and social work is of great significance in the practice of education.

According to Figure 3, it can be found that the crime rate of junior high school students is the highest, as high as 72%; the crime rate of high school students is the lowest, which is at 2%. When students receive education, it is not only the acquisition of knowledge but also the improvement and development of all aspects. They begin to learn and understand society and thus understand the inadmissibility of criminal behavior.

### 7.3. Current Situation and Problems of Youth Social Education

#### 7.3.1. Overall Status of Social Education in Our Country

Judging from the current status of social education development in various provinces and cities in our country, there are regional gaps in the development of youth social education. The cities with relatively developed economic infrastructure in the eastern coastal regions and the central region have carried out better social education for adolescents, while the western mountainous regions and the economically underdeveloped cities in the central region are less developed. The economic base determines the superstructure, and the relative underdevelopment of the economy results in the shortage of basic resources and teachers, which leads to the relative backwardness of social education.

### 7.4. Problems in Social Education

On the whole, youth education in our country is still in a superficial state, and the application of social work in education is relatively scattered, resulting in incomplete and unconcentrated social education. Through relevant data and analysis, the problems in social work can be summarized as shown in Figure 4.

#### 7.4.1. A Lack of Professional Talents and Not High Professional Quality

China's social work industry is in a positive stage of construction, and the industry's foundation is not enough. Therefore, only a part of the social education team has social worker qualification certificates. In this part of professional social workers, a considerable number of people lack social work experience and cannot effectively combine theory with practice, which has also led to the administration of social education for young people.

#### 7.4.2. The Not High Social Understanding of Social Work

The social work major is a subject newly added by universities in our country in a short time. In 1988, Peking University first opened the social work major, which only experienced short 30 years of construction in major universities. Therefore, when referring to the social work major, many people express that they do not understand the role of the subject or mistakenly understand the social work major as a profession engaged in community work in the future. These issues directly affect the social education of our youth. Social work is a sociology major. This major cultivates the professional values of “people-oriented, self-help, fairness, and justice,” that has a solid theoretical foundation, skilled social work methods, and other aspects of knowledge and ability and that can be used in party and government organs, enterprises, institutions and social organizations, and other departments and organizations. Compound application-oriented professionals are engaged in social work services and social welfare management in the field.

#### 7.4.3. The Not Perfect Relevant Laws and Regulations

Judging from the existing social education policies, the lack of relevant laws and regulations as support for social work intervention in social education has exacerbated the difficulty of combining social work with social education for youth.

From Figure 5, it can be seen that from 2008 to 2015, the number of documents with minors as keywords has gradually increased, reaching a maximum of 772 in 2015. In recent years, with the improvement of laws and regulations, the number of documents with minors as the key word has gradually decreased.

## 8. Strategies for Social Work Intervention

The essence of social work intervention in youth social education is to allow social workers to participate in social education activities, so the work can be divided into the following intervention areas, as shown in Figure 6.

### 8.1. Youth Field

The youth field means that according to the understanding of adolescents' physical and psychological characteristics, social workers combine with corresponding professional theoretical knowledge to promote the participation of young people in social education activities, such as summer camps, agricultural bases, agricultural bases, research activities, volunteer activities, and so on. Through these activities, youth groups can sum up the experience through their own experiences and gradually develop good habits so as to achieve the goal of comprehensive development of young people. The wide dissemination of social work among youth groups also promotes its development.

### 8.2. Family Field

The family plays an important role in the growth of teenagers. It can be said that the family is an individual enlightenment teacher. The participation of social workers in the family field refers to a way of living with young people to establish positive and harmonious family relationships, thereby realizing the support role of the family. According to the existing social work research and analysis of youth problems, it can be found that most of the youth problems are caused by negative family relationships. Therefore, promoting the construction of active family support is conducive to promoting the development of social education for young people.

### 8.3. School Field

School is the place with most adolescents, who spend most of their time on campus. Therefore, school work interventions have a positive effect on youth social education. For social work in schools, the principle of respect for students must be observed. Individuals are in the stage of thinking construction during adolescence, and immature thinking does not mean that teenagers have no standards for judging behavior. Therefore, in social work, people should regard adolescents as children or adults and maintain the principles of understanding and respect. At the same time, teachers should also pay attention to the help and interaction between students. In the classroom, teachers should pay attention to each student and actively exchange questions. After class, the teacher is the friend of the students and should pay attention to the emotional psychology of the students.

## 9. Conclusion

Youth is the hope of our country's future. The bad roots must be traced from the source, and the germ of juvenile crime must be eradicated from the source. A family is the assistant of society, the first that educates children. Parents are the enlightenment teachers, whose actions, words, and deeds have a subtle effect on the children. Intimate and harmonious family relationships and normal and good family education are crucial conditions for the healthy growth of every child. Every parent must have a full understanding of this and consciously assume a responsibility to society, which is also an essential part of reducing juvenile delinquency in society.

## Figures and Tables

**Figure 1:** Causes of juvenile cybercrime.

**Figure 2:** Prevention and control of juvenile cybercrime.

**Figure 3:** Crime rate.

**Figure 4:** Problems in social work.

**Figure 5:** Statistics on the number of documents with “minor” as the key word in 2008–2019.

**Figure 6:** Fields of social work involvement.

## Data Availability

This article does not cover data research. No data were used to support this study.

## References

[1] Meng L., Tu L. (2020). Research on the distribution and influencing factors of juvenile delinquency in my country. *Juvenile delinquency*.

[2] Chang J., Chen G. (2020). Structured theory: a new perspective on the causes of juvenile delinquency. *Research on Prevention of Juvenile Delinquency*.

[3] Meng F. (2020). Family environmental factors and correction of juvenile delinquency. *Legal System Expo*.

[4] Tan P. (2020). New characteristics of juvenile delinquency and analysis of its legal causes. *Legal System Expo*.

[5] Yuan S. (2020). Discussion on the new trends of juvenile delinquency and preventive measures. *Journal of Liaoning Police College*.

[6] Li Y. (2020). On starting with education to solve the psychological problems of young people. *Modern Enterprise*.

[7] Cui S. (2020). Systematic construction of prevention and control of juvenile delinquency in my country. *Journal of Heilongjiang Institute of Political and Legal Management Cadres*.

[8] Chang J. (2020). Space-time sociology: a new perspective on the causes of juvenile delinquency. *Chinese Youth Social Science*.

[9] Zhou X., Tang S., Cao J. (2019). Influencing factors and predictive analysis of juvenile delinquency in my country. *Legal System Expo*.

[10] Liu S. (2019). On the characteristics of current juvenile delinquency. *Legal System Expo*.

[11] Fu Z. (2019). Practice and thinking of social work intervention in juvenile crime correction——taking the pony case as an example. *Journal of Shandong Youth Politics College*.

[12] Guo Q. (2019). Sociological research on the causes of juvenile delinquency——from the perspective of family socialization function. *Office Business*.

[13] Liu C. (2019). Revision of the reverse psychological scale in criminal juveniles——a comparison of reverse psychology between ordinary and criminal teenagers. *Journal of Youth Studies*.

[14] Liu Y. (2019). The causes and preventive measures of juvenile delinquency under the current situation. *Legal System Expo*.

[15] Lv M. (2019). On the causes and countermeasures of juvenile delinquency. *Legal System and Society*.

[16] Zhang X. (2019). Thoughts on judicial social work involved in the family of criminals. *Society and Public Welfare*.

[17] Zhang G. (2019). Current situation and prevention of juvenile delinquency. *Crime Research*.

[18] Wang Y. (2019). Research and analysis of juvenile crime cases. *Legal System Expo*.

[19] Chen J. (2019). Analysis of the influencing factors of juvenile delinquency in my country. *Guilin University of Technology*.

[20] Zhang Y., Xin Y., Sun T. (2019). Investigation and analysis on the prevention patterns of juvenile delinquency and school violence. *Legal System and Society*.

[21] Zeng P., Chen J. (2019). Analysis of the influencing factors of juvenile delinquency in my country——an empirical study based on time series data. *Youth Research*.

[22] Yao Y. (2019). The causes and preventive measures of juvenile delinquency. *Journal of Changchun Education College*.

[23] Zhu P. (2019). The causes and countermeasures of juvenile cybercrime. *Modern Trade Industry*.

